The article "SERUM MUCOSA-ASSOCIATED EPITHELIAL CHEMOKINE IN ATOPIC DERMATITIS: A SPECIFIC MARKER FOR SEVERITY" was retracted in 2014. Reasons: duplicate publication; overlap with earlier publications.

# SERUM MUCOSA-ASSOCIATED EPITHELIAL CHEMOKINE IN ATOPIC DERMATITIS: A SPECIFIC MARKER FOR SEVERITY

**DOI:** 10.4103/0019-5154.55630

**Published:** 2009

**Authors:** M H M Ezzat, K Y Shaheen

**Affiliations:** *From the Department of Pediatrics, Faculty of Medicine, Ain Shams University, Cairo, Egypt.*; 1 *Department of Clinical Pathology, Faculty of Medicine, Ain Shams University, Cairo, Egypt.*

**Keywords:** *Atopy*, *CCL28*, *mucosa-associated epithelial chemokine*

## Abstract

**Background:**

Mucosa-associated epithelial chemokine (MEC; CCL28) is considered pivotal in mediating migration of CCR3 and CCR10-expressing skin-homing memory CLA^+^ T cells. CCL28 is selectively and continuously expressed by epidermal keratinocytes, but highly upregulated in inflammatory skin diseases such as atopic dermatitis (AD).

**Aims:**

This controlled longitudinal study was designed to evaluate the expression of CCL28 serum levels in childhood AD and bronchial asthma (BA) and its possible relations to disease severity and activity.

**Methods:**

Serum CCL28 levels were measured in 36 children with AD, 23 children with BA, and 14 children who had both conditions as well as in 21 healthy age and gender-matched subjects serving as controls. Sixteen patients in the AD group were followed-up and re-sampled for serum CCL28 after clinical remission. Serum CCL28 levels were correlated with some AD disease activity and severity variables.

**Results:**

Serum CCL28 levels in patients with AD whether during flare (median = 1530; mean ± SD = 1590.4 ± 724.3 pg/ml) or quiescence (median = 1477; mean ± SD = 1575.2 ± 522.1 pg/ml) were significantly higher than the values in healthy children (median = 301; mean ± SD = 189.6 ± 92.8 pg/ml). However, the levels during flare and quiescence were statistically comparable. The serum levels in BA (median = 340; mean ± SD = 201.6 ± 109.5 pg/ml) were significantly lower than the AD group and comparable with the healthy control values. Serum CCL28 levels in severe AD were significantly higher as compared with mild and moderate cases and correlated positively to the calculated severity scores (LSS and SCORAD). CCL28 levels during exacerbation of AD could be positively correlated to the corresponding values during remission, the peripheral absolute eosinophil counts, and the serum lactate dehydrogenase levels. Serum CCL28 did not vary with the serum total IgE values in AD.

**Conclusion:**

Our data reinforce the concept that CCL28 might share in the pathogenesis of AD probably through selective migration and infiltration of effector/memory Th2 cells into the skin. It may also represent an objective prognostic marker for disease severity. Further studies may pave the way for CCL28 antagonism among the adjuvant therapeutic strategies.

## Introduction

Atopic dermatitis (AD) is a common chronic inflammatory skin disorder of unknown etiology expressed early in life with peak incidence in early childhood. Disease development is primarily determined by as yet unknown genetic factors leading to the accumulation of peripheral activated T lymphocytes in the skin. It was hypothesized that AD is associated with an unbalanced establishment of the peripheral T-lymphocyte system. Cutaneous lymphocyte-associated antigen (CLA)[1] is a cell surface glycoprotein that has been postulated to play an important role in T-cell migration and homing to the skin. It has been proposed that interaction between T cells and epidermal keratinocytes plays a central role in the pathogenesis of AD.[2]

Mucosa-associated Epithelial Chemokine (MEC or CCL28) is a CC chemokine that has been recently identified and characterized and is a functional ligand for CC chemokine receptor-3 and 10 (CCR3 and 10). CCL28 gene is located on chromosome 5, and the corresponding cDNA encodes a 127 amino acid (AA) precursor protein with a putative 22 AA signal sequence. The signal sequence is cleaved to generate the 105 AA mature protein. Among human chemokines, CCL28 is most similar to the cutaneous T cell-attracting chemokine (CTACK or CCL27), with which is shares 40% AA identity.[3]

CCL28 has been reported to chemoattract transfectants expressing the seven-transmembrane G-protein coupled CCR3 and CCR10. Desensitization experiments had confirmed CCR10 specificity. CCR10, previously known as orphan G-protein-coupled receptor (GPR-2), has been detected on the surface of T lymphocytes, dermal microvascular endothelial cells, and dermal fibroblasts, but mRNA expression studies suggest that it may be present on additional cell types. CCL28 induces calcium mobilization in human CCR10-expressing transfectants by CCL27, indicating that these chemokines share the new receptor, CCR10.[4]

CCL28 is expressed in a wide range of human cell types and tissues. It appears to be predominantly produced by epithelial cells. Its mRNA expression is most abundant in salivary and mammary glands, human saliva, and breast milk.[5] Significant mRNA expression has also been observed in other tissues associated with mucosal epithelial surfaces, including the stomach, colon, rectum, nose, and trachea. The IL-10-/- knock-out mice display increased CCL28 expression in the stomach and Peyer's patches indicating that IL-10 may be CCL28 suppressive.[6] Studies showing CCL28 production in nasal and bronchial epithelial cell lines have suggested that it might also play a role in allergic respiratory diseases such as bronchial asthma (BA).

To our knowledge, there are no clinical studies on serum CCL28 levels in allergic diseases in the pediatric age groups to date. Also, no data on CCL28 levels in other biological fluid of allergic children could be cited in literature. Therefore, this study was conducted to explore the expression of CCL28 in AD and BA, hence its pathogenic role in such diseases to identify the clinical relevance of measuring serum CCL28 in terms of disease activity and/or severity.

## Materials and Methods

This follow-up controlled study was conducted over a period of 9 months from the first of January to the end of September 2005. All patients were enrolled from the Pediatric Allergy and Immunology Unit and outpatient clinic of the Ain Shams University Children's Hospital in Cairo. Informed consent was obtained from the parents or caregivers of each child before enrollment. Children were divided into the following three groups:

### Atopic dermatitis

This group comprised 36 children with AD diagnosed by standardized diagnostic criteria.[7] Their ages ranged between 8 and 120 months (mean ± SD = 47 ± 22 months). The group consisted of 20 males (55.5%) and 16 females (44.5%). The parents were subjected to a questionnaire concerning the precipitating factor(s). A possible cause could be traced in 18 children being exposed to food allergens [egg (6), milk (5), banana (4), and fish (3)]. In 18 children, the cause was not clear. For convenience, the severity of AD was evaluated according to two scores. First, the Leicester Sign Score (LSS; range = 0 to 108) in which severity is scored by 6 clinical features (erythema, purulence, excoriation/crusting, dryness/scaling, cracking/fissuring, and lichenification) graded at 6 defined body sites on a scale of 0 (none) to 3 (severe).[8,9] Second, the Scoring Atopic Dermatitis (SCORAD) index system that was used to evaluate the severity of eczema. This index includes the evaluation of extent, intensity, and subjective symptoms to a maximum score of 103 points.[10] Children with AD were classified into 3 groups (mild, moderate, and severe) according to a proposal for severity grading of AD using only objective criteria (mild AD, SCORAD score <15; moderate AD, score = 15-40; and severe AD, score >40).[11] Sixteen children (44.5%) presented with severe AD, 11 children (30.5%) presented with moderate severity, and 9 children (25%) were categorized as having mild illness. In the 16 patients with severe AD, serum CCL28 levels were measured before and after treatment with topical corticosteroids in combination with oral antihistamines. The response to treatment was scored using the Physician's Global Assessment (PGA) score. The PGA is an overall assessment from 0 to 5 of a patient's eczema, taking into consideration the quality and extent of lesions relative to the baseline assessment [0 = clear (100%), 1 = almost clear (90% to 99% improvement), 2 = marked improvement (50% to 89%), 3 = modest improvement (<50%), 4 = no change, and 5 = worse]. A total of 22 patients had AD only. The remaining 14 children had concomitant asthma (personal history and/or clinical evidences of respiratory allergy).

### Bronchial asthma

This group comprised 23 children enrolled while presenting with an acute asthmatic exacerbation. Their ages ranged between 14 and 90 months (mean ± SD = 49 ± 16 months). The group consisted of 12 males (52%) and 11 females (48%). From the patients' medical history, the asthma exacerbations were triggered by exposure to allergens (food, animal allergens, or both) in 12 children and upper respiratory tract infections in 5 children. In 6 children, the triggering agent was not clear. Ten children (43.5%) presented with acute severe asthma and the remaining 13 children (56.5%) presented with acute exacerbations of mild to moderate severity based on clinical data and peak expiratory flowmetry (PEFR).[12,13]

### Control group

This group comprised 21 healthy children without current or family history of allergic disorders. There were 12 males (57%) and 9 females (43%) in this group. Their ages ranged between 12 and 120 months with a mean ± SD of 77 ± 26 months. They underwent clinical examination to exclude any concomitant illness particularly allergic disorders and parasitic infestations. Children with peripheral blood eosinophilia or elevated serum IgE for their age were excluded.[14]

## Study Measurements

### Blood sampling

A total of 4 ml of venous blood was collected under complete aseptic conditions from each patient or control subject and was divided into 2 equal parts. One sample was mixed with EDTA as an anticoagulant for blood counting and the other was left to clot for 30 minutes for serum CCL28 assay. After coagulation, the latter sample was centrifuged for 15 minutes at 1000 × g. The separated sera were divided into 3 aliquots and stored at −20°C for the subsequent assay of serum CCL28, lactate dehydrogenase (LDH), and total IgE. Repeated thawing and freezing was avoided. Hemolyzed samples were excluded.

### Serum CCL28/MEC assay

The kit used was a human CCL28 immunoassay (Quantikine RandD Systems, Inc. McKinley Place N.E., Minneapolis, Minnesota 55413 U.S.A.). This assay employs the quantitative sandwich enzyme immunoassay technique using *E. coli*-expressed recombinant human CCL28 and antibodies raised against the recombinant factor. Results obtained using natural human CCL28 showed linear curves that were parallel to the standard curves obtained using the Quantikine kit standards.

A monoclonal antibody specific for CCL28 has been pre-coated onto a microplate. Standards and samples were pipetted into the wells and any CCL28 present was bound by the immobilized antibody. After washing away any unbound substances, a horseradish peroxidase-linked monoclonal antibody specific for CCL28 was added to the wells. Following a wash to remove any unbound antibody-enzyme reagent, a substrate solution of hydrogen peroxide-tetramethylbenzidine was added to the wells and color developed in proportion to the amount of CCL28 bound in the initial step. The color development was stopped by 2N sulfuric acid and the intensity of the color was measured at 450 nm and 540 nm. Readings at 540 nm were subtracted. For calculation of results, a standard curve was constructed on a log/log scale by plotting the mean absorbance for each standard on the y-axis against the concentration on the x-axis and drawing a best fit curve through the points on the graph. The minimum detectable dose (MDD) ranged from 0.58-6.05 pg/mL. The mean MDD was 2.58 pg/mL.

### Serum total IgE assay

This was performed in all subjects by quantitative enzyme immunoassay (Medix Biotech, San Carlos, CA, U.S.A.). Results were expressed in IU/ml. Owing to the variability in serum total IgE levels with age in childhood, we calculated the percentage values from the reference ranges by dividing the subject's actual level by the highest normal for age multiplied by 100.[14] IgE levels used in the correlations were both the measured and the calculated percentage values. The serum total IgE level that exceeded the highest normal for age was considered elevated.

### Complete blood count

A Coulter counter (Coulter MicroDiff 18, Fullerton, CA, U.S.A.) was used in this study. The differential leukocytic counts were estimated manually from the blood film and expressed in absolute count values. Infants and children whose absolute eosinophil counts (AEC) exceeded the normal reference values for age were considered to have peripheral blood eosinophilia. Blood sampling of all subjects was performed at the same time (10 am) daily to avoid diurnal variations in eosinophil counts.[14]

### Serum total lactate dehydrogenase assay

Serum total lactate dehydrogenase (LDH) (U/L) was measured only in the AD group during flare and in the healthy subjects. LDH assay was performed on an automatic chemistry analyzer (Synchron CX5 system, Beckman, Inc., Fullerton, CA, U.S.A.).

### Statistical analysis

All statistical analysis of the data was carried out using Statistical Package for the Social Science (SPSS), Version 9.02 for Windows^®^. Data were expressed as mean, standard deviation (SD), median, and interquartile ranges IQR (25^th^ and 75^th^ percentiles). A Student's *t* test was used for comparing parametric data. For non parametric comparison of serum CCL28 among different groups, a Mann-Whitney U test was used. The relation between the various numerical parameters was studied by the Pearson correlation coefficient (r) test with graphic representation using a linear regression line; r value was considered weak if < 0.5, moderate if ranged between 0.5-0.75, and strong if > 0.75. *P*-values below 0.05 for all tests were considered significant.

## Results

### Serum CCL28 levels of the studied groups

Serum CCL28 levels for patients with AD during a flare ranged between 687 and 2256 pg/ml (median = 1530, mean ± SD = 1590.4 ± 724.3 pg/ml) [Table 1]. These values were statistically comparable with the corresponding values of the same patients during quiescence, which ranged from 970 to 1980 pg/ml (median = 1477, mean ± SD = 1575.2 ± 522.1 pg/ml) (Z = 1.1; *P* > 0.05). The healthy children had much lower serum CCL28 levels (range = 10 to 460 pg/ml, median = 301, mean ± SD = 189.6 ± 92.8 pg/ml) as compared with the patients' data whether during flare (Z = 4.1; *P* < 0.0001) or quiescence (Z = 3.7; *P* < 0.0001) [Figure 1].

**Table 1:** Serum mucosa-associated epithelial chemokine in the study groups

Serum MEC/CCL28 (pg/ml)	AD		BA (flare)	AD + BA (flare)	Control group
				
	Flare	Quiescence			
Range	687-2256	970-1980	153-620	832-2059	10-460
Median	1530	1477	340	1425	301
IQR	1032	640	240	785	220
Mean	1590.4	1575.2	201.6	1601	189.6
SD	724.3	522.1	109.5	428.3	92.8
Z1	1.1	-	-	-	-
Z2	3.1*	2.9*	-	-	-
Z3	0.7	0.9	-	-	-
Z4	-	-	2.9*	-	-
Z5	4.1*	3.7*	0.4	3.9*	-

AD = Atopic dermatitis; BA = Bronchial asthma; IQR = Interquartile range; MEC = Mucosa-associated epithelial chemokine; SD = Standard deviation; Mann-Whitney test results: Z1 = AD flare versus quiescence; Z2 = AD versus BA; Z3 = AD versus (both AD and BA); Z4 = BA versus (both AD and BA); Z5 = Patients versus controls;

* = Highly significant (*P* < 0.0001)

**Figure 1:** Box-plot summary of serum mucosa-associated epithelial chemokine (MEC/CCL28) levels (pg/ml) in atopic dermatitis and control subjects (A Mann–Whitney test was used in the comparisons. Black squares represent the median and the boxes encompass the interquartiles (25^th^ and 75^th^ percentiles). The ranges are marked as maximum and minimum)

Serum CCL28 levels of asthmatic patients during exacerbations ranged between 153 and 620 pg/ml (median = 340, mean ± SD = 201.6 ± 109.5 pg/ml). These values were statistically comparable to the values of controls (Z = 0.4; *P* > 0.05), but were significantly lower than the values of children with AD whether during flare (Z = 3.1; *P* < 0.0001) or quiescence (Z = 2.9; *P* < 0.0001) [Figure 2].

**Figure 2:** A box-plot summary of serum mucosa-associated epithelial chemokine (MEC/CCL28) levels (pg/ml) in the study groups (A Mann–Whitney test was used in the comparisons)

Within the group of patients with AD, 14 subjects had concomitant asthma as well. Their serum CCL28 levels ranged from 832 to 2059 pg/ml (median = 1425, mean ± SD = 1601 ± 428.3 pg/ml). These values were statistically comparable with the values of the patients from the AD only group whether during flare (Z = 0.7; *P* > 0.05) or quiescence (Z = 0.9; *P* > 0.05), but were significantly higher when compared with the values of subjects with BA only (Z = 2.9; *P* < 0.0001) [Figure 2] and the control group (Z = 3.9; *P* < 0.0001).

### Serum CCL28 levels in relation to other clinical and laboratory variables

In our study, the mean SCORAD score values ranged between 10 and 65 (mean ± SD = 24.8 ± 10.6). The median and mean ± SD of serum CCL28 levels int he severe group (1809; 1754.8 ± 1110 pg/mL) were significantly higher than the corresponding values of the mild group (759; 785.1 ± 153.3 pg/ml; Z = 2.5; *P* < 0.001) or the moderate group (1190; 1165.9 ± 586.5 pg/ml; Z = 1.8; *P* < 0.01). Similarly, moderate cases had significantly higher values than the mild cases [Figure 3]. Moreover, serum CCL28 levels correlated positively with the LSS score and the SCORAD index (r = 0.89 and 0.70 respectively, *P* < 0.001 for both) [Figure 4], indicating CCL28 overexpression with increased severity.

**Figure 3:** A box-plot summary of serum mucosa-associated epithelial chemokine (MEC/CCL28) level (pg/ml) variations according to the atopic dermatitis SCORAD index of severity (A Mann–Whitney test was used in the comparisons.)

**Figure 4:** Serum mucosa-associated epithelial chemokine (MEC/CCL28) levels (pg/ml) in relation to atopic dermatitis severity scores; (a) the LSS and (b) the SCORAD index

A positive correlation could be elicited between the CCL28 serum levels during AD exacerbation and the corresponding values during remission meaning that the higher the level during acute attacks, the higher it remained after remission (r = 0.91; *P* < 0.0001) [Figure 5].

**Figure 5:** Positive correlation between the atopic dermatitis flare and remission levels of serum CCL28 (pg/ml)

The mean ± SD absolute eosinophil count values were statistically comparable among subjects with AD, BA, and AD associated with BA (650 ± 235, 590 ± 197, and 660 ± 301 cells/mm^3^, respectively). However, each value was significantly higher when compared with the control group (220 ± 90 cells/mm^3^; *P* < 0.01 for all groups). Serum CCL28 levels correlated positively with the absolute eosinophil count in all groups during flare (r = 0.73; 0.42 and 0.65, respectively; *P* < 0.01). A similar correlation was found in the AD group during quiescence (r = 0.87; *P* < 0.01). Another positive correlation could be elicited between the SCORAD index and the absolute eosinophil count in the AD group (r = 0.46; *P* < 0.05).

The studied patient groups (AD, BA, and AD associated with BA) were statistically comparable in terms of serum IgE levels (500.6 ± 385.6, 655 ± 492.5, and 627.9 ± 336.6 IU/ml, respectively) and each mean value was significantly higher than that of the healthy control subjects (140.6 ± 19.7 IU/ml; *P* < 0.001). Serum CCL28 or SCORAD index values could not be related by correlation coefficient to IgE concentrations or IgE percent values from normal in the studied groups.

Serum total LDH levels of patients with AD during a flare ranged between 130 and 1450 U/L (mean ± SD = 1036.6 ± 486.2 U/L). These values were significantly higher than the control values (range = 40–110 U/L; mean ± SD = 70 ± 25 U/L, *t* = 1.2; *P* < 0.05). LDH values correlated positively with each of the serum CCL28 levels and the SCORAD indices [Figure 6].

**Figure 6:** Positive correlations between serum total lactate dehydrogenase (LDH) (U/L) and serum CCL28 (pg/ml) (a) and the SCORAD index (b) in atopic dermatitis during flare

Serum CCL28 levels could not be correlated to age, weight centiles, and height centiles of subjects in each group. CCL28 expression was not influenced by age, gender, or family history. In the asthma group, CCL28 levels did not vary according to the PEFR values of patients.

## Discussion

MEC or CCL28 has been implicated in the homing of lymphocytes to the inflammatory sites. It was assumed to play an important role in T-cell migration to skin in adults with AD, psoriasis vulgaris, and bullous pemphigoid;[15] however, the expression of CCL28 in both normal children and children with atopic diseases has not been extensively studied. To evaluate a possible role of CCL28 estimation in pediatric allergy, we measured serum CCL28 levels in phenotypically well-defined groups of allergic children (AD, BA, and AD associated with BA) in comparison with a group of healthy non atopic age and gender-matched control subjects.

We observed that serum CCL28 levels were specifically elevated in patients with AD irrespective of allergic respiratory comorbidity. The study revealed that the levels in AD whether during a flare or exacerbation were significantly higher than the control group [Figure 1] and the asthmatic group [Figure 2]. Our results, which conform with those of Kagami, *et al*.,[15] probably reflect the upregulation of CCL28 in AD presenting a potentially useful marker for the presence of an atopic reaction. CCL28 regulation by allergen exposure and microbial products suggests an important role for CCL28 in the initiation and amplification of the atopic skin response. The failure to demonstrate a significant reduction in serum CCL28 levels after remission of the flare [Figure 1] could be due to the ongoing process of subclinical allergic cutaneous inflammation. Also, it could be indicative of the need for more intensive non conventional anti-inflammatory therapy. Therefore, we suggest that serum CCL28 levels be used as a marker for the ongoing inflammatory activity in the skin.

Among human chemokines, CTACK (CCL27) is most similar to MEC (or CCL28) sharing 40% AA identity.[3] Like CCL28, CCL27 is also known to recruit CLA^+^ memory Th2 lymphocytes.[16] Dose-dependent chemotaxis of identical lymphocyte populations in response to CCL28 is nearly indistinguishable from that exhibited by CCL27; except that CCL28 has higher maximal activity.[17,18] CCL27 was found to be expressed at high levels in the epidermis of lesional skin biopsy specimens from patients with AD compared with non lesional skin.[19,20] Owing to the tissue-specific expression profile and receptor specificity of both chemokines (CCL27 and CCL28), a definite role of CCL28 in AD is highly suggested.

CCL28 is expressed in a variety of human tissues, and it appears to be predominantly produced by epithelial cells.[5] It is strongly expressed constitutively in lesional epidermal keratinocytes of patients with AD and psoriasis vulgaris.[15] *In vitro*, CCL28 displays chemotactic activity for resting CD4^+^ CD8^+^ T cells.[4] These cells can be detected in a significant proportion in the peripheral blood of children with AD.[1] This may suggest a faulty maturation of the T-lymphocyte system as a basic pathophysiological change in AD, leading to skin inflammation with CD4^+^ CD8^+^ T lymphocytes resembling immature T cells.[21] This is likely to lead to the skewing of many immune reactions in those patients.

CCL28 is also displayed by cutaneous venules and is strongly expressed on endothelial cells. It is thought that it triggers vascular arrest of circulating skin homing memory T cells, which uniformly express CCR10, particularly CLA^+^ CCR10^+^ memory T cells. Chronic cutaneous inflammation induces CD4^+^ T cells expressing E-selectin binding activity in draining lymph nodes. CLA is a ligand for E-selectin, an adhesion molecule, which is critical in recruiting T cells. These E-selectin ligand^+^ T cells migrate efficiently to CCL28 and to CCL27 as well.[22,23]

This could reinforce the hypothesis that CCL28 and CCL27 may work in a sequential way, with CCL28 acting mainly in the first steps of T-cell recruitment by inducing integrin-dependent adhesion and transendothelial migration of T cells and CCL27 playing a major role in the migration of T cells into the upper layers of the skin. Finally, T cells infiltrating the epidermis may result in the induction of apoptosis in keratinocytes, resulting in spongiosis, which is the histologic hallmark of eczema.

To test the specificity of CCL28 response in AD, we sought to investigate its expression in a group of subjects with asthma during acute exacerbations. The serum CCL28 levels of patients with asthma were statistically comparable to the values of controls, but were significantly lower as compared with the values of children with AD whether during flare or quiescence. The normal values of serum CCL28 in our patients with asthma indicates that the results of studies that use bronchial cell lines and mouse models[24,25] cannot simply be extrapolated to human studies *in vivo*. It is also possible that the local production of CCL28 in mucosal epithelial cells may be insufficient to lead to a systemic increase.

In children who presented with concomitant allergic cutaneous and respiratory diseases (BA and AD), the overexpression of CCL28 can be ascribed to the presence of AD, supporting further evidence for the implication of CCL28 in atopic cutaneous responses. Our data may thus reflect the upregulation of CCL28 in AD specifically; however, our findings are still limited by the sample size.

Serum CCL28 levels in subjects categorized as severe AD cases were significantly higher as compared with the moderate and mild groups with a positive correlation to the LSS and SCORAD severity scores [Figures 3 and 4]. This substantiates the usefulness of this parameter as a skin-specific objective marker of disease severity in AD.

A large variety of laboratory measurements[26,27] have been linked to disease activity and severity in AD, however most of them lack specificity.

The high levels of IgE in AD have not been satisfactorily explained but can be ascribed to a deficiency of IgE isotype-specific “suppressor” T-cell function. It has not been established that AD is exclusively an IgE-mediated allergic disorder; and it is difficult to demonstrate consistently a role for allergens in the pathogenesis. Although patients with AD frequently possess IgE antibody specific for inhalants or food allergens, it is not generally possible to induce skin lesions or AD by intradermal injection of the suspected allergen.[28,29] Moreover, typical lesions of AD may occur in individuals with X-linked agammaglobulinemia who have virtually no IgE.[7]

Serum CCL28 levels and the SCORAD score results in the current study could not be correlated to the serum total IgE concentrations or percent values from normal during AD flare. Our results were not concordant with some reports.[27,28] The discrepancy can be ascribed to the small number of cases with elevated IgE category (6 children only). We also recruited subjects at different stages of disease activity and serum total IgE levels are known to fluctuate throughout the disease stages.

On the other hand, serum CCL28 concentrations and the SCORAD indices correlated positively with the absolute eosinophil counts both during AD flare and quiescence. Previous studies had identified eosinophil chemoattractant properties of CCL28 using human cells.[4,24] It is not clear whether CCL28 may have a role in regulating the constitutive numbers of eosinophils in peripheral blood by inducing eosinophil chemotaxis in a CCR3 and CCR10-dependent manner. Animal studies confirmed that CCL28 was a chemoattractant for murine eosinophils. There appears to be a temporal relationship of CCL28 production with eotaxin and other CCR3 ligands in animal models.[24] Perhaps they play an important role for the localization of eosinophils around the inflammatory sites. Interestingly, anti-CCL28-treated animals also showed reduced eosinophil accumulation.[30] Therefore, we might conclude that CCL28, a CCR3 ligand, is important for various stages of eosinophil migration and/or activation within tissues. It might be possible one day to target tissue eosinophilia in severe allergic diseases by manipulating CCL28/CCR3 interactions.

The serum total LDH levels of our patients with AD during flare were significantly higher as compared with controls. Moreover, significant positive correlations could be elicited between serum LDH levels during flare and serum CCL28 concentrations and SCORAD indices [Figure 6]. Elevated levels can be attributed to its release from damaged lesional epidermal cells into peripheral blood reflecting the extent of skin involvement and the degree of epidermal injury. LDH was previously reported as useful yet it was not a specific marker for severity of skin eruption being elevated in many other diseases.[31,32]

In conclusion, it seems that serum CCL28 expression is upregulated in children with AD irrespective of allergic respiratory comorbidity. It might be one of the important chemokines in the lesional formation of AD and might have a distinct role in the development of atopy/allergy skin phenotypes. It could be a useful specific inflammatory marker for assessing AD severity in children. Further research using immunohistochemical staining of CCL28 in the lesional AD skin and other cutaneous hypersensitivities are warranted as well as studies addressing the relations between its expression and the conventional lines of treatment used. A potential role of CCL28 in respiratory allergy deserves further evaluation on a wider scale. Moreover, the effect of CCL28 antagonists and other immunotherapeutics, like monoclonal antibodies on the CCL28 kinetics is worth evaluation. CCL28 antagonism may provide a conceptual basis for the development of new therapeutic strategies in cases of severe AD.
